This article has been retracted.

# METTL3 Accelerates Breast Cancer Progression via Regulating EZH2 m^6^A Modification

**DOI:** 10.1155/2022/5794422

**Published:** 2022-03-29

**Authors:** Shaojun Hu, Yang Song, Yu Zhou, Yu Jiao, Guopeng Li

**Affiliations:** ^1^Department of Oncological Surgery, First Affiliated Hospital of Jiamusi University, Jiamusi, China; ^2^Department of Pathology, First Affiliated Hospital of Jiamusi University, Jiamusi, China; ^3^Department of General Surgery, The First Hospital of Qiqihar, Qiqihar, China; ^4^Department of General Surgery, Affiliated Qiqihar Hospital, Southern Medical University, Qiqihar, China

## Abstract

We aimed to investigate the bio-functions of METTL3 in promoting breast cancer (BCa) progression via regulating N6-methyladenosine (m^6^A) modification of EZH2 mRNA. METTL3 levels in 48 cases of BCa and matched paracancerous tissues were detected. In the meantime, METTL3 in BCa patients with different staging or lymphatic metastasis states were examined. Prognosis of the BCa patients was analyzed using Kaplan–Meier estimator. Protein levels of EMT-associated genes and invasive and migratory abilities were evaluated. The binding relationship between EZH2 and METTL3 was analyzed via RIP. Besides, m^6^A modification of EZH2 mRNA was explored. E-Cadherin level in MCF-7 cells with EZH2 knockdown was tested. Subsequently, ChIP was done to verify the interaction between E-cadherin and EZH2. Regulatory effects of METTL3/E-cadherin axis on EMT and metastasis of BCa were finally determined. METTL3 was upregulated in BCa tissues compared to paracancerous ones. METTL3 was especially higher in T3-T4 BCa or those with lymphatic metastasis. BCa patients expressing high level of METTL3 experienced worse survival. METTL3 was identically upregulated in BCa cell lines. Knockdown of METTL3 in MCF-7 cells attenuated EMT and metastatic abilities. Protein level of EZH2 was downregulated after knockdown of METTL3 in MCF-7 cells, while its mRNA level was not influenced by METTL3. Furthermore, METTL3 was confirmed to interact with EZH2, and m^6^A modification existed in EZH2 mRNA. Knockdown of EZH2 greatly upregulated mRNA level of E-cadherin, and later, ChIP assay confirmed the interaction between EZH2 and E-cadherin. E-Cadherin could abolish the effects of METTL3 on BCa metastasis and epithelial-mesenchymal transition. METTL3 is upregulated in BCa. It could regulate the protein level of EZH2 through m^6^A modification to promote EMT and metastasis in BCa cells, thereafter aggravating the progression of BCa.

## 1. Introduction

As the highest prevalent malignancy in females, breast cancer (BCa) accounts for nearly 24.2% of all kinds of cancers, and its death cases account for 15% [1, 2]. In China, the newly onset and tumor death cases of BCa account for 12.2% and 9.6%, respectively [3]. Surgical procedures and target therapies for BCa have achieved great progressions. Nevertheless, tumor recurrence, metastasis, and drug-resistance of BCa severely affect the prognosis [4–7].

N6-methyladenosine (m^6^A) modification is a kind of common RNA modification in eukaryotic mRNAs [8]. RNA translation efficiency, RNA degradation, subcellular localization, alternative splicing, etc., are all influenced by m6A [9–12]. METTL3 maintains the homeostasis of m6A methylation by methylation of its target mRNAs. It extensively participates in tumor diseases [13–15]. However, the molecular mechanism of METTL3 in BCa development remains still unclear.

Enhancer of zeste homolog 2 (EZH2) inhibits the expressions of tumor-suppressor genes [16]. Moreover, after downregulation of METTL3, its reduction inhibited both H3K27me3 and EZH2 [17]. However, whether a similar mechanism exists in breast cancer is unclear. Epithelial-mesenchymal transition (EMT) is a common processing where the morphology and function of epithelial cells transform to those of mesenchymal cells [18–23]. In BCa, EMT triggers tumor cells to migrate and invade, thus resulting in local infiltration and distant metastasis [24–26].

This study analyzed the potential function of METTL3 in inducing m^6^A modification of EZH2, thereafter influencing the malignant progression of BCa.

## 2. Materials and Methods

### 2.1. Samples

Primary BCa (*n* = 48) and paracancerous tissues (*n* = 48) were collected from our hospital. The age of all patients range from 41 to 83 years old and median age was 67. None of the BCa patients received preoperative antitumor therapy. BCa tissues and paracancerous ones were obtained, and pathological stages were evaluated by an experienced pathologist in our hospital. This study was approved by the Ethics Committee of First Affiliated Hospital of Jiamusi University and also got the signed written contents from the patients/family members. The clinic-pathological details of clinical samples are shown in Table 1.

### 2.2. Cell Transfection

BCa cells (MCF10A, MCF-7, and BT474) were washed, digested, and centrifuged. Cell transfection was conducted by Lipofectamine 2000 according to the instructions from the manufacturer.

### 2.3. Quantitative Real-Time Polymerase Chain Reaction (qRT-PCR)

TRIzol was used to extract the total RNA. *qRT-PCR* was conducted according to previously established instructions. GAPDH and U6 were considered as the internal references. Relative level was quantified using 2^−ΔΔCt^ method. The primer sequences used are shown in Table 2.

### 2.4. Western Blotting

The total protein extracted from the cells was quantified via bicinchoninic acid method. Protein samples with the adjusted same concentration were separated and then loaded on polyvinylidene fluoride membranes followed by being blocked with defatted milk (5%) for 2 hours and then incubated with primary antibodies (GAPDH: cat#AF5009, METTL3: cat#ab195352, E-cadherin: cat#ab76055, N-cadherin: cat#ab18208, vimentin: cat#ab92547, and *α*-SMA: cat#ab108424) at 4°C overnight. Thereafter, secondary antibodies were applied for further incubation for 2 h followed by bands being exposed via ECL kit.

### 2.5. Transwell Assay

Matrigel was diluted with serum-free medium after thawed overnight at 4°C. The membrane coated with diluted Matrigel at the basolateral chamber was then dried at room temperature. 3 × 10^4^ cells were inoculated on the top of a Transwell insert placed in a 24-well plate. 100 *μ*L of serum-free medium was applied in the bottom. After 24 hours of incubation, cells infiltrated to the bottom were soaked in the methanol for 15 min, stained using crystal violet for 20 min, and counted microscopically. For migration assays, the cells were seeded and format in wells without Matrigel precoating in the inner side of each insert. Invasion and migration abilities were accessed through counting the number of cells invaded through the Matrigel and migrated into the basolateral chamber.

### 2.6. RNA-Binding Protein Immunoprecipitation (RIP) and Chromatin Immunoprecipitation (ChIP) Experiments

The corresponding antibodies or anti-IgG were used for incubation of the cells overnight at 4°C. The protein-RNA complex is obtained after the antibody captures the intracellular specific protein. The protein was then digested with proteinase K and the RNA was extracted. The immunoprecipitant RNA was finally subjected to qRT-PCR for determining the relative level. ChIP was conducted using the kit. Chromatin immunoprecipitated DNA was eluted, reversely X-linked, purified, and subjected for qRT-PCR.

### 2.7. Statistical Analyses

GraphPad Prism and Statistical Product and Service Solutions 18.0 were employed for data analysis. Comparisons between multiple groups were performed using one-way ANOVA test followed by least significant difference as its post hoc test. Statistical significance was set as *P* < 0.05.

## 3. Results

### 3.1. METTL3 Was Upregulated in BCa and Predicted Poor Prognosis

METTL3 levels in BCa and paracancerous tissues were first detected. METTL3 was markedly upregulated in BCa tissues (Figures 1(a) and 1(b) and Table 1). Notably, METTL3 was higher in T3-T4 BCa than that of T1-T2 (Figure 1(c), Table 1). BCa patients with lymphatic metastasis expressed higher abundance of METTL3 relative to nonmetastatic patients (Figure 1(d), Table 1). We also found that the expression of METTL3 BCa patients with tumors ≤2 CM was significantly higher than that >2 CM (Table 1). Through analyzing follow-up data of enrolled BCa patients, Kaplan–Meier results demonstrated worse prognosis in BCa patients with high expressed levels of METTL3 (Figure 1(e)).

### 3.2. Knockdown of METTL3 Blocked EMT and Metastasis in BCa

Compared with human normal mammary epithelial cells MCF10A, METTL3 was highly expressed in BCa cells MCF-7 and BT474 (Figure 2(a)). We also determined that the protein levels of METTL3 in MCF-7 and BT474 were higher than in MCF10A (Figure 2(b)). Since the patients in this study were all estrogen receptors (ER) (+), but not all patients were progesterone receptors (PR) (+), we chose the MCF-7 cell line for subsequent research. Subsequently, METTL3 mRNA and protein levels were effectively knocked down by transfection of si-METTL3 in MCF-7 cells (Figures 2(c) and 2(d)). EMT-related proteins were detected by western blotting. It was demonstrated that E-cadherin was upregulated, while N-cadherin, vimentin, and *α*-SMA were downregulated after si-METTL3 transfection in MCF-7 cells (Figure 2(e)). Transwell experiments depicted attenuated invasive and migratory abilities in MCF-7 cells with si-METTL3 (Figure 2(f)). As a result, METTL3 was able to induce EMT and stimulate metastasis in BCa.

### 3.3. METTL3 Regulated m^6^A Modification of EZH2

EZH2 protein was markedly downregulated by si-METTL3 in MCF-7 cells (Figure 3(a)). It is speculated that there may be a potential interaction between EZH2 and METTL3. As RIP assay results demonstrated, EZH2 was remarkably enriched in anti-METTL3 (Figure 3(b)). Meanwhile, the presence of m^6^A modification was found in EZH2 mRNA (Figure 3(c)). Interestingly, qRT-PCR data illustrated that transfection of si-METTL3 has not affected EZH2 mRNA in MCF-7 cell lines (Figure 3(d)). The above findings suggested that METTL3 regulated protein level of EZH2 through m^6^A modification of EZH2 mRNA.

### 3.4. METTL3 Downregulated E-Cadherin through EZH2 Recruitment and Thus Promoted Malignancy of BCa

EZH2 siRNA (si-EZH2) was prepared for further clarifying the function of EZH2 in BCa. Transfection of si-EZH2 markedly downregulated EZH2 (Figures 4(a) and 4(b)) and upregulated E-cadherin (Figures 4(c) and 4(d)) in MCF-7 cells. Subsequently, ChIP experiment confirmed that EZH2 can bind to E-cadherin promoter region, thus silencing its expression (Figure 4(e)). It is shown that knockdown of E-cadherin could reverse protein level changes of E-cadherin, N-cadherin, and vimentin in MCF-7 cell lines with si-METTL3 (Figure 4(f)). Moreover, knockdown METTL3 decreased the cell migration and invasion, but the attenuated metastatic abilities of MCF-7 cells with METTL3 knockdown were partially reversed by knockdown of E-cadherin (Figure 4(g)). As a result, E-cadherin was responsible for malignant progression of BCa regulated by METTL3 through EZH2 recruitment.

## 4. Discussion

Tumorigenesis originates from alterations on oncogenes and tumor-suppressor genes, thereafter leading to protein dysregulation and carcinogen activation [27]. Evidence has shown that METTL3 was able to accelerate the proliferation, migration, and invasion of cancer cells via posttranscriptional modification [28]. METTL3 was also reported to play an important role in the development of gliomas by increasing glioma stem-like cell (GSC) maintenance and radioresistance [29]. The current study demonstrated that METTL3 was significantly upregulated in BCa tissues than that of paracancerous tissues. METTL3 was especially higher in T3-T4 BCa or those with lymphatic metastasis. BCa patients with high expressed METTL3 levels experienced worse survival. Results also showed that METTL3 was involved in the progression of BCa.

It is reported that m^6^A modification was involved in the regulation of gene expressions through affecting translation efficiency and splicing [30, 31]. A recent study showed that m^6^A modification influences histone modifications [32]. In this paper, knockdown METTL3 increased the E-cadherin and decreased the N-cadherin and vimentin, indicating that METTL3 promoted the progress of EMT. Moreover, we also noticed that after METTL3 was knocked down, the protein level of EZH2 was reduced, but its mRNA level was not significantly changed, indicating that METTL3 has a posttranscriptional modification of EZH2. METTL3 regulated protein level of EZH2 by mediating the m^6^A modification of EZH2, thus affecting EMT and malignancy of BCa cells.

EZH2 is a histone-lysine methyltransferase containing 751 amino acids and it is located on human chromosome 7q35 [33]. As an important component of catalytic complex of PRC2, EZH2 catalyzes H3K27me3 and silences target genes [34–36]. Our findings showed that knockdown of METTL3 in MCF-7 cells attenuated EMT and metastatic abilities. Only protein level of EZH2 was downregulated after knockdown of METTL3 in MCF-7 cells, while its mRNA level remained unchangeable. Furthermore, METTL3 was confirmed to interact with EZH2, and m^6^A modification existed in EZH2. Knockdown of EZH2 greatly upregulated mRNA level of E-cadherin, and later, ChIP assay confirmed the interaction between EZH2 and E-cadherin. Notably, E-cadherin could abolish the effects of METTL3 on BCa metastasis and EMT. Collectively, METTL3 induced EMT in BCa via m^6^A modification of EZH2 mRNA.

METTL3 is upregulated in BCa. It could regulate protein level of EZH2 through m^6^A modification to promote EMT and metastasis in BCa cells, thereafter accelerating BCa progression.

## Figures and Tables

**Figure 1:** METTL3 was upregulated in BCa and predicted poor prognosis. (a) METTL3 mRNA levels in BCa tissues and paracancerous ones. (b) METTL3 protein levels in BCa tissues and paracancerous ones. (c) METTL3 levels in BCa patients with T1-T2 or T3-T4. (d) METTL3 levels in BCa patients either with lymphatic metastasis or not. (e) The overall survivals in 2 groups of BCa patients.

**Figure 2:** Knockdown of METTL3 blocked EMT and metastasis in BCa. (a) qRT-PCR detected the METTL3 mRNA levels, (b) western blotting determined the METTL3 protein expressions in MCF10A, MCF-7, and BT474 cells. (c, d) si-METTL3 was used to know-down the mRNA and protein levels of METTL3 in MCF-7 cells. (e) E-Cadherin, N-cadherin, vimentin, and *α*-SMA were measured via western blotting in MCF-7 cells transfected with NC or si-METTL3. (f) Migration and invasion in MCF-7 cells transfected with si-METTL3.

**Figure 3:** METTL3 regulated m^6^A modification of EZH2. (a) Western blotting detected EZH2 protein level in MCF-7 cells transfected with NC or si-METTL3. (b) EZH2 enrichment in anti-METTL3, input, or anti-IgG group. (c) EZH2 enrichment in input, m^6^A, or anti-IgG. (d) The mRNA level of EZH2 in MCF-7 cells transfected with si-METTL3.

**Figure 4:** METTL3 downregulated E-cadherin through EZH2 recruitment and thus promoted malignancy of BCa. (a) qRT-PCR detected the METTL3 mRNA levels; (b) western blotting determined the METTL3 protein in MCF-7 cells transfected with si-EZH2; (c) qRT-PCR detected E-cadherin mRNA levels; (d) western blotting determined E-cadherin protein in MCF-7 cells transfected with si-EZH2; (e) E-cadherin enrichment in anti-IgG, anti-EZH2, or anti-H3K27me3; (f) protein levels of E-cadherin, N-cadherin, and vimentin in MCF-7 cells transfected with si-METTL3 or si-METTL3 + si-E-cadherin; (g) migration and invasion in MCF-7 cells transfected with si-METTL3 or si-METTL3 + si-E-cadherin.

**Table 1:** The demographic data of the enrolled patients (*n* = 48).

Items	*N*	Low-METTL3 (*n* = 24)	High-METTL3 (*n* = 24)	*P* value
Age (*y*)				
≤50	23	11	12	0.7726
>50	25	13	12	
Tumor size				
≤2 CM	25	17	8	0.0093^*∗*^
>2 CM	23	7	16	
TNM staging
I∼II	28	19	9	0.0034^*∗*^
III∼IV	20	5	15	
Lymph node metastasis				
No	25	18	7	0.0015^*∗*^
Yes	23	6	17	

^∗^ *P* < 0.01.

**Table 2:** Primer sequences.

Gene	Primer sequences
EZH2	F: 5′-TGCACATCCTGACTTCTGTG-3′
	R: 5′-AAGGGCATTCACCAACTCC-3′

E-ca	F: 5′-AAAGGCCCATTTCCTAAAAACCT-3′
	R: 5′-TGCGTTCTCTATCCAGAGGCT-3′

METTL3	F: 5′-AGATGGGGTAGAAAGCCTCCT-3′
	R: 5′-TGGTCAGCATAGGTTACAAGAGT-3′

GAPDH	F: 5′-CGGAGTCAACGGATTTGGTCGT-3′
	R: 5′-GGGAAGGATCTGTCTCTGACC-3′

## Data Availability

The raw data supporting the conclusions of this article will be made available by the authors, without undue reservation.
